# Small cell lung cancer progressing into fatal ascending motor and sensory polyneuropathy despite dramatic response to chemotherapy: A case report

**DOI:** 10.1097/MD.0000000000041172

**Published:** 2025-01-03

**Authors:** Syed Mohammad Naqvi, Hashim Talib Hashim, Syed Yaseen Naqvi, Ahmed Qasim Mohammed Alhatemi, Fatimah Abdullah Sulaiman, Sally Muayad Abdulmahdi, Ahmed Dheyaa Al-Obaidi, Ashraf Fhed Mohammed Basalilah, Ammar Al-Obaidi

**Affiliations:** a National Institute for Prevention and Cardiovascular Health (NIPC), University of Galway, Galway, Ireland; b College of Medicine, University of Warith Al-Anbiyaa, Karbala, Iraq; c Department of Internal Medicine, Al-Nassiryah Teaching Hospital, Nassiryah, Thi Qar, Iraq; d Radiology Techniques Department, College of Health and Medical Techniques, Al-Mustaqbal University, Babylon, Iraq; e College of Medicine, University of Baghdad, Baghdad, Iraq; f Department of Internal Medicine, Hadhramaut Hospital, Hadhramaut, Yemen; g Department of Hematology/Oncology, University of Missouri-Kansas City, Kansas, MO.

**Keywords:** cancer, dramatic response to chemotherapy, fatal ascending motor and sensory polyneuropathy, oncology, small cell lung cancer

## Abstract

**Rationale:**

Paraneoplastic syndromes occur in 10% to 20% of all malignancies, with paraneoplastic neurological syndromes in less than 1% of all malignancies. In small cell lung cancer (SCLC), paraneoplastic manifestations are more common, affecting up to 5% of cases. Common manifestations include syndrome of inappropriate antidiuretic hormone secretion, Cushing’s syndrome due to adrenocorticotropic hormone secretion, paraneoplastic cerebellar degeneration, and Lambert-Eaton myasthenic syndrome. Paraneoplastic acute motor and sensory polyneuropathy is an exceptionally rare but severe complication, necessitating timely diagnosis and management.

**Patient concerns:**

A 55-year-old male with an 80 pack-year history of smoking presents to the hospital with a 3-week history of fevers, productive cough, dyspnoea, and wheeze. He had no significant comorbidities.

**Diagnoses:**

Extensive radiological investigations revealed a large mass at the right hilum compressing on the right lower bronchus with metastatic adrenal deposits. Biochemical investigations confirmed syndrome of inappropriate antidiuretic hormone secretion, and histology identified SCLC.

**Interventions:**

Despite initiating a combination chemotherapy with carboplatin and etoposide, the patient developed progressive motor paralysis and sensory loss over 4 days, leading to a diagnosis of paraneoplastic acute motor and sensory polyneuropathy.

**Outcomes:**

He deteriorated rapidly and died 14 days after symptom onset due to respiratory failure, underscoring the aggressive nature of paraneoplastic syndromes.

**Lessons:**

Paraneoplastic syndromes, particularly in SCLC, pose significant diagnostic and therapeutic challenges. This case highlights the importance of early recognition and prompt multidisciplinary intervention, which may improve outcomes despite the low incidence of these severe complications. Treating cancer with appropriate systemic chemotherapy or suppression of the immune response alleviates neurological symptoms and improves prognosis.

## 1. Introduction

Small cell lung cancer (SCLC) constitutes 15% of all lung cancers. It commonly occurs in heavy smokers. Its aggressive nature results in surgery having a limited role. Commonly regarded as a systemic disease at presentation, a minority present with limited stage disease. In limited stage disease, platinum-based chemotherapy regimens in combination with concurrent thoracic radiotherapy offers a possibility of long-term disease-free survival. Rates of metastatic disease are high with up to 20% harboring the risk of brain metastasis at presentation or during the course of the disease.^[1]^ For patients with extensive stage disease, doublet platinum-based chemotherapy remains the standard of care for those with preserved functional performance status. Radiotherapy is reserved in these cases for palliation or symptom control. Other alternatives include single agent chemotherapy such as topotecan or taxanes.

Paraneoplastic syndromes are rare, occurring in 10% to 20% of all malignancies. Paraneoplastic neurological syndromes (PNS) occur in <1% of all malignancies. However, in the setting of SCLC paraneoplastic syndromes can occur more frequently and up to 5% of cases develop PNS. More common paraneoplastic manifestations of SCLC can include inappropriate antidiuretic hormone secretion (SIADH), adrenocorticotropic hormone secretion causing Cushing’s syndrome, paraneoplastic cerebellar degeneration and Lambert–Eaton myasthenic syndrome.

Neurological symptoms in patients with SCLC could be due to several causes including malignant central nervous system involvement, chemotherapy-induced neuropathy (most commonly presenting as peripheral sensory neuropathy secondary to cisplatin or paclitaxel) or less commonly albeit well documented, paraneoplastic phenomenon. There are few case reports of SCLC initially presenting as ascending paralysis or later becoming apparent during the course of chemotherapy. We herein describe a case of SCLC with paraneoplastic SIADH at diagnosis, which later becomes complicated by fatal ascending motor and sensory neuropathy.

This case report is significant due to its unique combination of features: the rapid progression of paraneoplastic motor and sensory polyneuropathy associated with SCLC, atypical electrophysiological findings, and the dissociation between the oncological and neurological responses to treatment. While paraneoplastic syndromes are rare, occurring in 3% to 5% of SCLC cases, this case emphasizes the importance of early recognition and intervention to manage these potentially fatal complications effectively.

## 2. Case presentation

A previously well, 55-year-old male was referred to emergency department by his family doctor complaining of a 3-week history of fevers, productive cough, dyspnea and wheeze. He had an 80-pack year smoking history and a positive family history of lung cancer. He had been treated by his family doctor with a course of oral amoxicillin and oral prednisone, but his symptoms deteriorated. On presentation to emergency department his white cell count was 16.4 × 109/L (normal range: 4.0–10.0 × 109/L) neutrophil count of 13.8 × 109/L (normal range: 2.0–7.0 × 109/L), C-reactive protein was 118 mg/L (normal 0–5 mg/L) and serum sodium was 112 mmol/L (normal range: 136–145 mmol/L). Other biochemical markers were within normal limits. A chest X-ray showed right middle and lower lobe consolidation with associated moderate pleural effusion (Fig. 1). He was admitted and treated as community acquired pneumonia and work-up confirmed SIADH.

**Figure 1.** Chest X-ray of the patients.

The patient deteriorated despite intravenous Piperacillin–Tazobactam and oral Clarithromycin with worsening of consolidation on repeat chest X-ray. The patient was transferred to the intensive care unit and subsequently intubated and ventilated. A computerized tomography (CT) scan of his thorax revealed a right hilar mass with mediastinal involvement and right-sided hilar adenopathy with superimposed extensive air space consolidation (Fig. 2). A biopsy performed during bronchoscopy revealed histologically monotonous, small cells with dark ovoid nuclei. No nucleoli were seen, and several mitotic figures were present. The cells have narrow ill-defined cytoplasm. Immunohistochemistry performed on the tumor cells showed CD45 negativity, AE1/AE3, TTF1 positivity. Focal minimal synaptophysin and chromogranin A positivity were also seen. This immunohistochemical profile was consistent with a diagnosis of small cell lung cancer.

**Figure 2.** CT scan of the thorax revealed a right hilar mass with mediastinal involvement and right-sided hilar adenopathy with superimposed extensive air space consolidation. CT = computed tomography.

Full staging consisting of a CT-scan of the brain and Thorax–Abdomen–Pelvis confirmed extensive stage disease with adrenal metastases. The patient’s ECOG performance status was poor due to a combination of the SCLC and respiratory distress warranting artificial ventilation. As response rates with chemotherapy in SCLC are generally high, chemotherapy doublet in the form of carboplatin and etoposide were commenced while the patient was intubated in the ICU.

The patient responded well to treatment and was extubated and transferred to the ward on noninvasive ventilation. A re-staging CT-Thorax after 1 cycle showed good partial response to treatment (Fig. 3).

**Figure 3.** Coronal-section CT-thorax on diagnosis (L) and after cycle 1 of chemotherapy (R). CT = computed tomography.

On cycle 2 day 3 of chemotherapy, the patient developed lower back pain and bilateral lower limb weakness. Examination identified bilateral lower limb motor (Medical Research Council [MRC] Grade 3) and sensory paresis. Sensory examination revealed absent light touch, pinprick, coordination and proprioception in the lower limbs. Day 3 of Etoposide was held as a result of the new neurological findings.

A CT-Brain, Magnetic Resonance Imaging (MRI)-Brain and MRI-spine were performed to investigate the new neurological findings. All radiology was reported as normal with no evidence of intracerebral metastases, stroke, myelitis or leptomeningeal disease. In addition, there was no obvious radiographic evidence of spinal cord compression either by extrinsic compression by osseous metastatic deposit or intramedullary or leptomeningneal deposits.

Two days later, a repeat neurological examination revealed tetraplegia, MRC Grade 0 in both upper and lower limbs. All deep tendon reflexes were absent. Head and neck muscles, cognition and speech were unaffected, and cranial nerve examination was normal.

Routine blood investigations including C-reactive protein and erythrocyte sedimentation rate were normal. Specific blood investigations including serum vitamin B12, folate, HIV serology, Lyme disease serology, Epstein-Barr virus serology, Brucella serology, thyroid antibodies, thyroid function tests, ANCA, ENA, ANA and serum protein electrophoresis were all negative or normal. Antibodies for Hu, Ri and Yo blood tests were sent, and all were negative. At this point a diagnosis of acute ascending motor and sensory symmetrical polyneuropathy was suspected and a lumbar puncture was performed. The results of cerebrospinal fluid (CSF) revealed an elevated total protein of 3.32 g/L (normal 0.15–0.45), and other parameters were normal, with a repeat 3 days later showing similar results. CSF cytology was negative for malignancy and CSF culture was also negative.

Electromyography was consistent with diffuse predominantly motor polyneuropathy; sensory potentials were preserved but they were of small amplitude. The motor conductions show mixed axonal/demyelinating features, which was not typical of Guillain–Barre Syndrome.

Electromyography and nerve conduction studies were conducted to investigate the patient’s acute motor and sensory polyneuropathy. The nerve conduction studies revealed the following:

• **Motor nerves:**
◦ Compound muscle action potential (CMAP) amplitudes were markedly reduced in the tibial and ulnar nerves bilaterally (tibial: 1.2 mV; normal > 4 mV; ulnar: 0.8 mV; normal > 3 mV).
◦ Motor conduction velocities (MCV) were slowed in the tibial and ulnar nerves (tibial: 30 m/s; normal > 40 m/s; ulnar: 34 m/s; normal > 50 m/s), consistent with demyelination.
◦ Distal motor latencies were prolonged, with a mixed axonal and demyelinating pattern.
• **Sensory nerves:**
◦ Sensory nerve action potential (SNAP) amplitudes were preserved but of small amplitude in the sural and median nerves (sural: 4 μV; normal > 10 μV; median: 6 μV; normal > 15 μV).
◦ Sensory conduction velocities (SCV) were within normal limits.

The electrophysiological findings revealed a predominantly motor polyneuropathy with mixed axonal and demyelinating features, atypical for classical paraneoplastic syndromes, which are generally sensory predominant and characterized by absent SNAPs.

In the interim, while these investigations were ongoing, the patient was started on intravenous dexamethasone and 0.4 g/kg/day of intravenous immunoglobulin without any symptomatic improvement.

## 3. Outcomes and follow up

Despite a significant initial oncological response to chemotherapy, the patient’s neurological condition deteriorated rapidly. Following 1 cycle of carboplatin and etoposide, imaging confirmed a partial response with a reduction in tumor size. However, the onset of severe, ascending motor and sensory polyneuropathy led to respiratory compromise. This dissociation between the oncological and neurological responses highlights the aggressive and refractory nature of PNS, even when cancer treatment is effective. Although intravenous dexamethasone and intravenous immunoglobulin were administered promptly, they failed to improve neurological outcomes.

Lengthy repeated multidisciplinary discussions were held with the patient and his family regarding further Intensive Care Unit admission for ventilatory support. The patient was well informed and aware that reversibility of his neurological symptoms was unlikely and therefore he opted for best supportive care. The patient subsequently died 3 weeks after initial symptoms. The patient’s decision to decline further invasive ventilatory support in favor of palliative care highlights the ethical considerations surrounding quality of life in rapidly progressive paraneoplastic syndromes.

## 4. Discussion

A paraneoplastic syndrome refers to cancer-associated signs and symptoms arising in organs and tissues that are remote from the cancer and unrelated to metastasis.^[2]^ Paraneoplastic syndromes are rare, affecting <1% of patients with cancer, and only 3% to 5% of cases of SCLC are affected.^[3]^ Most patients with these rare syndromes have high titers of antibodies against neuronal proteins that are abnormally expressed in SCLC tumors.^[4]^

Few case reports in the literature describe a coexistence of SCLC and Guillain–Barre like syndrome.^[5,6]^ Anti-Hu antibodies have a specificity of 99% and sensitivity of 82% in detecting paraneoplastic neurological syndrome, and SCLC is the underlying malignancy in more than 90% of cases.^[7]^ There are 2 approaches to treatment: the first is to treat the cancer with systemic treatment, the second is to suppress the immune reaction with the use of corticosteroids, intravenous immunoglobulin, plasma exchange, azathioprine or cyclophosphamide.^[7]^ Treatments of these syndromes are generally poor.

The patient’s respiratory failure was most likely attributable to the progression of paraneoplastic neuropathy rather than worsening of the malignancy. This conclusion is supported by the following observations:

- Imaging of the chest revealed a significant reduction in the hilar mass and mediastinal adenopathy postchemotherapy, indicative of a good oncological response. No evidence of recurrent or progressive tumor burden affecting the phrenic nerves or central respiratory control centers was identified.
- Neurological examination demonstrated preserved cranial nerve function, excluding brainstem involvement as a cause of respiratory insufficiency.
- The rapid development of diaphragmatic weakness in conjunction with the ascending motor paralysis aligns with severe motor neuropathy as the primary mechanism.

While diaphragmatic electromyography was not performed, the electrophysiological findings of widespread motor axonal dysfunction suggest a loss of lower motor neuron input to the respiratory muscles. This phenomenon has been reported in severe cases of paraneoplastic polyneuropathy associated with SCLC.

## 5. Study limitations

This case report has several limitations. First, while the clinical diagnosis of paraneoplastic acute motor and sensory polyneuropathy was supported by electrophysiological findings, the absence of specific anti-neuronal antibodies, such as anti-Hu, limits the definitive confirmation of a paraneoplastic etiology. Secondly, diaphragmatic electromyography was not performed, which could have provided direct evidence of respiratory muscle involvement. Additionally, the absence of postmortem examination precludes definitive exclusion of alternative pathologies, such as metastatic infiltration of the nervous system. Finally, as a single case report, generalizability to broader populations remains limited, necessitating caution when extrapolating these findings to other SCLC patients presenting with similar neurological complications.

## 6. Conclusion

This case underscores the critical importance of early recognition and management of PNS in SCLC. It highlights the complex duality in treating SCLC with paraneoplastic complications; while tumor reduction through chemotherapy can be successful, it does not always translate into improved overall prognosis when aggressive PNS are present. The dissociation between oncological success and neurological deterioration emphasizes the urgent need for early diagnosis and potentially more aggressive or innovative immunological interventions. Future research should focus on developing targeted therapies for paraneoplastic syndromes to enhance both survival and neurological outcomes in patients with SCLC.

## Author contributions

**Conceptualization:** Syed Mohammad Naqvi, Fatimah Abdullah Sulaiman, Ashraf Fhed Mohammed Basalilah.

**Data curation:** Syed Mohammad Naqvi, Fatimah Abdullah Sulaiman, Sally Muayad Abdulmahdi, Ammar Al-Obaidi.

**Formal analysis:** Syed Mohammad Naqvi.

**Funding acquisition:** Hashim Talib Hashim, Ammar Al-Obaidi.

**Investigation:** Hashim Talib Hashim, Syed Yaseen Naqvi, Fatimah Abdullah Sulaiman, Sally Muayad Abdulmahdi.

**Methodology:** Syed Yaseen Naqvi.

**Project administration:** Syed Yaseen Naqvi.

**Resources:** Ahmed Qasim Mohammed Alhatemi, Sally Muayad Abdulmahdi, Ahmed Dheyaa Al-Obaidi, Ashraf Fhed Mohammed Basalilah.

**Software:** Ahmed Dheyaa Al-Obaidi, Ashraf Fhed Mohammed Basalilah.

**Supervision:** Hashim Talib Hashim, Sally Muayad Abdulmahdi, Ammar Al-Obaidi.

**Validation:** Hashim Talib Hashim, Syed Yaseen Naqvi.

**Visualization:** Syed Yaseen Naqvi.

**Writing – original draft:** Hashim Talib Hashim, Syed Yaseen Naqvi, Ahmed Qasim Mohammed Alhatemi, Fatimah Abdullah Sulaiman, Ahmed Dheyaa Al-Obaidi, Ashraf Fhed Mohammed Basalilah.

**Writing – review & editing:** Syed Mohammad Naqvi, Ahmed Qasim Mohammed Alhatemi, Sally Muayad Abdulmahdi, Ammar Al-Obaidi.
